The article "Incentive mechanism of multiple green innovation behaviors of equipment manufacturing enterprises: A managers, green coordination groups and employees perspective" was retracted in 2025. Reasons: concerns about the results or conclusions; concerns about the peer review; concerns about the authorship.

# Incentive mechanism of multiple green innovation behaviors of equipment manufacturing enterprises: A managers, green coordination groups and employees perspective

**DOI:** 10.1371/journal.pone.0300533

**Published:** 2024-03-20

**Authors:** Baohong Li, Shi Yin, Baosheng Zhang

**Affiliations:** 1 School of Economics and Management, Harbin Normal University, Harbin, China; 2 School of Economics and Management, Harbin Engineering University, Harbin, China; 3 College of Economics and Management, Hebei Agricultural University, Baoding, China; Zhejiang Shuren University, CHINA

## Abstract

Employees play a pivotal role in the implementing of green development strategies and the attainment of dual-carbon objectives within manufacturing enterprises. Effective motivation of employees, fostering consensus on environmental protection, increased engagement in environmental initiatives, and the cultivation of employee cohesion are all vital for fostering green development within these enterprises. This paper seeks to elucidate the roles of general managers, green coordination groups (GCG), and employees in actualizing green behaviors. Furthermore, it advocates for a double incentive model to be employed in the implementing of green strategies within manufacturing enterprises. The research reveals that multiple factors, including incentive intensity, green capability, effort cost, risk aversion, and green variance, significantly influence the formulation of incentive contracts for green behaviors. The motivation level of the general manager directly impacts the efforts of the GCG, the organization’s green climate, the manager’s individual efforts, and indirectly influences the motivation and efforts of employees towards green behaviors. Notably, the influence of the organization’s green climate on employees surpasses than on the manager, underscoring the imperative for collaboration efforts between the general manager and GCG to instill green behaviors among employees. Hence, it is imperative for the general manager and GCG to collaborate not only on critical aspects of green strategy implementation but also in fostering green behaviors among employees. This collaboration will facilitate the development of a multi-layer incentive mechanism aimed at promoting and facilitating the adoption of green behaviors among employees, thus contributing to the advancement of theory regarding employees’ green behaviors and offering practical guidance for effectively realizing dual-carbon targets and achieving high-quality development within enterprises.

## 1. Introduction

Environmental problems such as climate change [1, 2], water pollution, and energy waste [3] pose a serious threat to the sustainable human development and have garnered global attention [4, 5]. Sustainable development has always been highly prioritized [6]. In September 2020, General Secretary Xi Jinping proposed that China would increase its independent national contribution to achieve carbon peak by 2030 and carbon neutrality by 2060. The double carbon goals set high demand for enterprises to achieve green development, meaning they must quickly surpass the gradual development process to achieve green and high-quality development in a short time [7].With the government green regulation combined with market demand for green products and services, enterprises have become the main battleground for energy saving and environmental protection. They must choose to implement specific green development goals to proactively balance production and operation activities with environmental protection; achieving economic and environmental benefits has become a top priority of enterprises [8].This includes initiatives such as utilizing renewable energy sources, reducing waste and emissions, and adhering to sustainable business practices. In this regard, scholars focus on how enterprises can attain high-quality green development [9]. For example, Zhang proposed a three-stage approach that combines an end-of-pipe governance green strategy, resource chain closed-loop green strategy, and three-chain super-loop green strategy [10]. However, concerning enterprises’ transition green practices[11], their green innovation behaviors are fundamental to the success of green strategy implementation [12, 13]. Stimulating green innovation behaviors among employees at all levels has become a new issue as enterprises aim for sustainable development and green strategies implement [14–16]. Improving the green behavior of employees is considered an crucial micro-activity for enterprises to achieve green and low-carbon development. Employees’ efforts in energy conservation, emission reduction, environmental protection, and resources recycling contribute and innovating green products, providing green services, establishing a green corporate image gaining green competitive advantages, and ultimately achieving higher economic performance. Therefore, deeply exploring the incentive problem of employees’ green behavior to effectively untilize internal resources, technology, information, and to obtain economic performance and environmental performance, holds significant significance.

Currently, scholars and businesses are increasingly focusing on research related to motivating employees’ green behavior. The research primarily emphasize the significance of executives’ environmental awareness and responsibility, the factors influencing employees’ green behavior, and methods for incentivizing such behavior. Zutshi and Sohal (2004) underscored the pivotal role of top management’s leadership and support in corporate environmental management [17]. They are tasked with appointing members to green coordination teams, overseeing environmental issues, providing leadership and motivation to employees at all levels, setting goals for green coordination teams, and evaluating performance. Meng et al. (2015) argued that executives’ environmental awareness and responsibility affect the formulation and implementation of corporate green strategies [18].Zou et al. (2019) suggested that executive cash compensation incentives encourage companies to adhere to green strategies and engage in green management practices [19].A study observed that many companies are beginning to motivate executives to achieve green and sustainable development goals [20].Cahan and Schweiger (1993) stressed the importance of integrating environmental, health, and safety (EHS) issues into corporate processes, asserting that green management is everyone’s responsibility in a company [21].Pujari (2004) emphasized the necessity of clear leadership and active support from executives in the industrial new product development process [22]. Kartadjumena and Rodgers noted that higher executive compensation motivates executives to exert more effort in addressing environmental issues, thereby improving corporate performance [23]. Zhao and Xiao(2021) discussed factors influencing employees’ green behavior, highlighting the influence of individual characteristics and green organizational culture [24]. Peng et al. (2018) examined the influence of an environmentally friendly organizational atmosphere on employees’ green behavior [25]. Zhou and Zhao (2023)proposed rewarding individuals, including employees and other stakeholders, for their implementation of green behaviors [26].

Despite limited research on incentive mechanisms for employees’ green behavior, both academic and practical realms recognize that achieving environmental goals in manufacturing enterprises necessitates collaboration at all organizational levels [27]. aligning employees’ green behavior with the company’s green strategic goals and fostering effective collaboration among employees are crucial for the successful implementation of green strategies [28].

While there has been extensive global research on incentivizing employees for green behavior, studies focusing on specific companies as research subjects are limited. In the current global context, changes in the world energy market, the impact of the COVID-19 pandemic, the shock of war [29–31],and the challenges of industrialization and urbanization [32] are imposing significant resource constraints on manufacturing enterprises. These enterprises are increasingly aware of their responsibility for green development, boosting green investments, and recognize the importance of green innovation. However, due to the large baseline of overall emissions, relatively weak green innovation, and the difficulty of replacing fossil fuels in the short term, achieving carbon neutrality remains challenging. To address this, manufacturing enterprises have established professional departments based on digital technology, agile management, and flat organizational models to coordinate and allocate enterprise resources, create a green organizational atmosphere, stimulate employees’ green behavior, and optimize the allocation of green resources. Examples include cross-departmental green product development departments, special peak carbon and carbon neutrality action groups, and joint project groups for carbon management systems [7].These entities, collectively known as Green Coordination Groups (GCG), play a crucial role in enhancing the effectiveness of manufacturing enterprises in implementing green strategies.

In the context of information asymmetry, the supervision of employees’ green behavior by general managers is costly and impractical, leading to the delegation of incentive measures and supervision of employees’ green behavior to the GCG. Consequently, the implementation of green strategies, improvement of environmental performance, and fulfillment of environmental responsibilities all involve dual agency relationships. Motivating coordination groups and employees to implement green behavior to achieve the green strategy of manufacturing enterprises is one of the most pressing challenges. The concept of dual agency is widely applied in incentivizing green behavior as it accurately describes the relationships involved. Existing studies rarely integrate the general manager-GCG-employee relationship into a single theoretical framework, thus failing to elucidate the dual agency relationship in the implementation of green strategies in manufacturing enterprises. Therefore, this paper aims to place these three types of green behaviors within the same incentive framework, specifically addressing the dual agency relationship and constructing a dual agency model that includes the general Manager-GCG-Employees. This paper analyzes factors such as incentive intensity, green capability, green cost coefficient, risk aversion, green variance, and organizational green atmosphere, exploring the operating mechanism of the incentive model. Its purpose is to provide a theoretical basis and practical experience for promoting the implementation of corporate green strategies.

The remainder of this study is structured as follows. Section 2 provides a comprehensive literature review. Section 3 outlines the model construction and its corresponding solution. Section 4 presents the results. Section 5 includes a detailed numerical analysis. Section 6 offers the study’s conclusion and practical implications. Lastly, Section 7 discusses limitations and suggests future perspectives.

## 2. Literature reviews

### 2.1 Research related to green innovation

In recent years, there has been a growing emphasis on green development in research. Key areas of interest including government regulation [33],the empowering of green technology [34],various green manufacturing models [35], and technological innovation in the green sector [36–39]. Wu et al. (2022) investigate the impact of government-led green publicity on corporate green behavior in China, providing empirical evidence on the relationship between government-led initiatives and corporate environmental behavior [40]. Zhu et al.(2023) developed a tripartite evolutionary game model for governments, demonstration enterprises, and small to medium-sized manufacturing enterprises, proposing a governance mechanism for digital transformation strategy [33]. In the context of digital empowerment of green development, Xue et al. (2022) explored the potential of digital transformation in promoting green technology innovation, shedding light on the role of digital technologies in fostering sustainability [41]. Feroz et al.(2021) emphasized the need for comprehensive studies to understand the impacts of digital transformation on environmental sustainability, highlighting the importance of considering the impact on corporate social responsibility and environmental performance [42]. Ren et al. (2023) focused on the impact of the digital economy on the green transformation of China’s manufacturing industry, providing empirical evidence of how digital technologies promote green transformation through technological innovation and industrial structure optimization [43]. Zhu et al. (2024) explored the application of blockchain technology in low-carbon supply chains and its influence on strategies for reducing carbon emissions. Factors such as consumer trust, low-carbon preferences, brand awareness, blockchain operation and construction costs, as well as the research and development difficulty of reducing carbon emissions, were considered [34]. Concerning green manufacturing models, Zhu et al. (2023) proposed that green manufacturing is a crucial measures for energy conservation and emission reduction. They introduced three green manufacturing models: the product remanufacturing model, green product manufacturing model, and hybrid manufacturing model [35]. In the realm of green innovation, Abdul-Rashid et al. (2017)explored the impact of sustainable manufacturing practices on sustainability performance, underlining the significance of these practices in preserving the environment and enhancing human life quality during manufacturing activitie [44]. Additionally, Zhu et al. (2023)studied the impact of altruistic preferences on carbon emissions on e-commerce platforms, developing "cost-sharing" contracts to enhance carbon emission reduction levels in the electronic supply chain and among manufacturers [39].Some literature confirms the positive impact of green innovation on corporate environmental performance [45–47]. Most industries achieve improved corporate environmental performance by reducing energy intensity, enhancing resource utilization efficiency [48]. These studies provide a solid theoretical and practical foundation for the green development of enterprises at the technological and strategic levels. However, there exists a research gap in the micro-mechanisms of implementation and management of green strategies, especially concerning the dynamics involving managers, green coordination teams, and employee behavior. Consequently, scholars have shifted their focus to researching the implementation and management of green strategies, involving Senior Management, Green Coordination Teams, and Employee Green Behavior. Cai et al. (2023) emphasize that the green development of enterprises depends not only on business strategies and technologies but also on the transformation of management models and incentive mechanisms, requiring the collaborative efforts of senior management, middle management, and general employees [49]. Additionally, Shah and Soomro (2023) highlight the necessity for alignment between corporate green strategies and employee green behaviors for the successful implementation of such strategies [28].

### 2.2 Research related to motivating employees toward green innovation behaviors

Regarding research on senior management’s green incentives and influence: Recent studies have shifted their focus towards examining the green behaviors exhibited by corporate executives [16]and employees [30],recognizing their pivotal roles in facilitating corporate green transformation. Cai et al. (2023) delved into how green servant leadership can effectively stimulate voluntary green behaviors among employees, leveraging informal mechanisms such as value orientation and cultural atmosphere [49].Empirical findings by Wu and Tham (2023) highlight the positive impact of providing green incentives to senior managers on a company’s environmental, social, and governance (ESG) performance [50]. The transformation leadership abilities of CEOs [51] and the influence exerted by senior management’s green behaviors on corporate green perceptions [52] have been identified as crucial factors. It’s evident that the green incentives extended to senior managers play a pivotal role in steering organizations towards sustainable development and augmenting corporate value. Simultaneously, research pertaining to motivations and incentives for employee green behavior has primarily focused on individual factors such as green motivation [53], green attitudes [54], green commitment, along with situational factors including colleague support, green organizational climate [55], and human resource management practices, and their collective impact on fostering employee green behavior. These investigations underscore the positive influence by these factors on employee engagement in green practices [56]. Furthermore, emphasis has been placed on the significance of cultivating a green organizational climate in facilitating the implementation and management of corporate green strategies [57].A conducive green organizational climate encompasses internal policies, practices, and values that advocate sustainability and environmentally friendly behaviors [58]. Such a positive climate not only enhances employee satisfaction, engagement, and organizational commitment but also instills a sense of pride and purpose among employees [25], as they perceive themselves as contributing to a larger cause beyond their individual job responsibilities. Overall, a supportive green organizational climate serves as a catalyst for encouraging employee participation in green initiatives.

Despite the existing research conducted on the green behaviors of executives and employees, there remains a gap in the literature concerning green behaviors across various managerial levels–encompassing general managers, middle managers, and employees–under the same incentive structure. Given that the formulation and execution of green strategies are iterative and collaborative endeavors, further comprehensive investigation is warranted into the underlying motivations driving employee green behaviors, especially in the context of dual-target objectives implementation.

### 2.3 Research related to double principal-agent theory

Dual Agency Theory expands upon traditional principal-agent relationships by incorporating an intermediary who serves as the agent in the initial layer and as the principal in the subsequent layer. This theory delves deeply into the dynamics among the three parties, with the aim of formulating an optimal contract that satisfies the conditions of all parties involved, thereby maximizing the utility of the dual agency actors. Scholars worldwide have extensively studied this theory, primarily focusing on its practical feasibility and applications across various domains. The research encompasses topics such as audit collusion among auditors [59], the contextual factors and advantageous conditions conducive to the emergence of dual agency [60]and the dual agency relationships between major shareholders and managers, as well as between major and minor shareholders [61, 62].Moreover, the multi-layered principal-agent relationships among shareholders, the government, and management in state-owned enterprises [63] underscore the superiority of the dual agency model over the single-layered model. This offers both theoretical and practical significance for developing green incentive mechanisms. In recent years, scholars have increasingly explored incentive issues related to corporate green behavior within the framework of dual agency theory. Case studies have examined the application of dual agency relationships among governments, corporations, and executives in promoting green objectives [16], as well as the application and oversight of green technology by central and local governments and corporations [64]. Furthermore, addition has been drawn to employee behavior incentive mechanisms based on Dual Agency Theory, including knowledge-based employee innovation incentive mechanisms, reputation mechanisms, and multi-task principal-agent models [65].Studies have also analyzed employees’ decision-making processes and performance differences in innovative behaviors within the framework of incentive mechanisms [66]. In the implementation of green strategies, the general manager, GCG, and employees play crucial as key executors [67].Their actions in green product design, green production, green marketing, and green recycling significantly influence the green performance of manufacturing enterprises. Therefore, fostering a positive green organizational atmosphere, reducing the effort cost, and appropriately rewarding and penalizing green behaviors among employees are crucial for improving their green behavior. The question of how to motivate green behaviors to enhance a company’s [68] environmental performance remains a topic worthy of further exploration.

This study, grounded in Dual Agency Theory, investigates the implementation of green strategies in manufacturing enterprises, with a specific focus on the roles and functions of three key agents involved in promoting green behavior: the general manager, the Green Coordination Group (GCG), and the employees. By situating these agents within a unified incentive framework and considering the crucial contextual factor of organizational green atmosphere, the research aims to explore the development of contract-based incentive mechanisms. These mechanisms are crafted not only to motivate the general manager in leading the GCG in green management and coordination but also to motivate the green coordination team to further incentivize employees across departments to implement green strategies. Additionally, the study examines the interrelationships among these agents, providing theoretical insights and practical guidance for enhancing green behaviors among employees in manufacturing enterprises.

The paper makes significant contributions in three key areas: Firstly, it advances research on employee green behavior by expanding the investigation scope to include incentives. Utilizing dual principal-agent theory, it explores the roles of the general manager, green coordination team, and employees in driving green strategies, addressing a gap in existing literature. Secondly, it enriches the application of principal-agent theory by recognizing the dual role of the green coordination team in modern manufacturing. It proposes a model involving the general manager, coordination team, and employees, shedding light on incentivizing environmentally responsible behaviors. Lastly, it provides theoretical and simulation evidence for constructing incentive systems, emphasizing collaboration between the general manager and coordination team. Factors like incentive intensity, green capability, and effort cost coefficient are identified as crucial in designing effective incentive contracts, essential for sustainable development in equipment manufacturing enterprises.

## 3. Methodology

### 3.1 Analysis of double principal-agent relationships in the implementation of green strategies

In navigating the complexity of implementing green strategic objectives, multiple actors are involved with intricate interconnections. This paper concentrates on three pivotal levels: the general manager, the Green Coordination Group (GCG), and the employees. These levels are critical in realizing the enterprise’s green strategic objectives, as delineated in the referenced literature [64].This focused approach simplifies the research, enabling a clearer understanding of the dynamics at play in achieving these environmental goals.

In the pursuit of implementing green strategic objectives, various actors are engaged, and the interconnections among them are intricate. To streamline this research, the paper centers its focus on three key levels essential to the implementation of the enterprise’s green strategic objectives: the general manager, the Green Coordination Group (GCG), and the employees.

Specifically, the implementation of the green strategy involves two distinct levels. Firstly, it is encompasses the principal-agent relationship existing between the general manager and the GCG. Secondly, it encompasses the principal-agent relationship between GCG and employees across various departments. The role of general manager at the forefront is crucial; tasked with driving efficiency and effectiveness toward achieving the double carbon targets [69]. In the short-term, the focus lies on meeting national energy-saving and environmental protection requirements, while aiming for relevant national and international green certification in the longer term. These efforts culminate in the establishment of core competitiveness within the green market. The position of the general manager holds weight as it symbolizes the enterprise’s dedication to green development. Acting as the company’s senior manager, the general manager’s actions serve as a reflection of the company’s green strategy. Externally, the general manager’s alignment with green value profoundly impacts the company’s ability to proactively implement green strategies, establish a green image, and secure market share within the green sector. Internally, the general manager plays a crucial role in spearheading the formation of Green Coordination Group (GCG),nurturing a green organizational culture, and reshaping incentive mechanisms.

The green behaviors of the general manager include:(1)In the context of the double carbon strategy, the general manager plays a pivotal role in establishing targets for energy conservation and environmental protection [70, 71]. This encompasses the selection of a green value creation model, the coordination of green resources and the assurance of competitive advantage. These actions are integral to ensuring the successful implementation of strategy, thereby securing both economic and environmental benefits for the enterprise.(2)The general manager delegates the responsibility of attaining the double carbon target to the GCG. Concurrently, they formulate management incentive contracts aimed at maximizing returns.(3)In their leadership role, the general manager cultivates employees’ green values by promoting positive environmental attitudes and integrates these values into their daily work routines.(4)The general manager assesses and oversees the green output results of the enterprise.

Tian (2022)advocates for the establishment of green action teams within enterprise [72]. Building on this, Yang and Liu (2010) propose the formation of a green action group, tasked with coordinating and overseeing initiatives related to energy conservation reduction. This group is instrumental in implementing the green action plan of enterprises [73]. Acting as an intermediary principal, the GCG assumes the responsibility of formulating policies and regulations for energy conservation and environmental protection. This strategic approach is designed economic benefits and showcase the organization’s managerial prowess.

The objectives of the GCG’s initiative encompass several key aspects:(1)Cultivating a green organizational atmosphere conducive to sustainable development.(2)Enhancing employee consciousness regarding environmental responsibilities.(3)Streamlining the coordinating and allocating green resources.(4)Furnishing requisite institutional, organizational, and personnel support for the environmentally-friendly transformation of pivotal production elements.(5)Crafting motivational contracts for employees, with an emphasis on career planning and development, and incentivizing green behaviors.(6)Facilitating green training programs to augment employees’ proficiency in low-carbon initiatives, disseminating knowledge on sustainable practices, and stimulating engagement in low-carbon green innovation [74, 75].

In its intermediary role, the GCG assumes dual identities:

1. As an agent, it may leverage informational asymmetries to circumvent regulations and advances its own interests, particularly in scenarios where oversight by the general manager is insufficient.
2. As a principal, it could demonstrate inertia, posing challenges to the establishment of a mechanism ensuring the sustained implementation of the double carbon targets.

Significantly, the GCG, in its role as the executor of dual carbon targets, does not possess ownership of the assets and thus does not reap benefit from asset appreciation. This absence of direct incentives can diminish motivation to promote staff involvement and present an agency risk.

The employees, positioned as end agents, operates under the directives and oversight of both the general manager and the GCG to execute energy-saving and emission-reduction initiatives. These employees comprises diverse roles, encompassing R&D personnel dedicated to green technology advancement, front line production staff, data analysts tasked with mining customer data to address environmental demands, and green marketing professionals. Notably production line employees exemplify this commitment by spearheading innovation across product design, manufacturing, and sales processes. For instance, they anticipate that embracing green innovation will not only boost productivity but also yield increase economic returns. Motivated by the prospect of amplifying their individual contribution, employees leverage their expertise in exploring and propose innovations, with a focus on optimizing process technology, equipment maintenance, and reconfiguration of production processes [76].

In the implementing of the green strategy, the general manager, the GCG, and the employees occupy distinct management levels, hold diverse roles, and consequently pursue varying objectives, albeit with the overarching goal of maximize their individual interests. However, owing to information asymmetries, the general manager faces challenges in accurately assessing the GCG’s efforts in coordinating resource allocation and motivating employees. Similarly, the GCG encounters difficulty in precisely evaluating the employees’ contributions to energy conservation and emission reduction. This asymmetry creates potential risks of moral hazard and adverse selection, as both the GCG and employees, acting as agents, may exploit their informational advantage for personal gain. To mitigate these risks, the general manager optimizes green performance by designing incentive contracts for the GCG. Subsequently the GCG, seeks to maximize desired outcomes by formulating incentive contracts for the employees, who, in turn, enhance their certainty-equivalent returns through their green, low-carbon actions. For a more comprehensive, refer to Fig 1.

**Fig 1:** The double principal-agent model in the implementation of enterprise the green strategy.

### 3.2 Model assumptions and parameter descriptions

Assumption 1: Risk-neutral for the general manager, risk-averse for managers and employees[72], and Arrow–Pratt Absolute risk aversion; *ρ*_1_, *ρ*_2_(>0) [73].

Assumption 2: The environmental performance output of employees who practice green innovation behaviors in all parts of the production process of an enterprise is mainly related to their own efforts and their ability to behave greenly. Therefore, the linear function of an employee’s current green innovation behaviors performance is *π*_2_ = *λ*_2_*e*_2_ where *λ*_2_(*λ*_2_>0) represents the ability of employees to act greenly (employee commitment, education level, attitude towards the environment).

The GCG helps to implement the company’s double carbon green targets by coordinating resources and motivating staff through green management capabilities. The general manager needs to motivate the GCG based on their management capability, effort, and dedication to creating a green atmosphere in the organization. A linear function of the manager’s ability to demonstrate performance through green management is $\pi_{1}=\lambda_{1}e_{1}+\theta_{1}+\eta (\lambda_{2}e_{2}+\theta_{2})$ where *λ*_1_(*λ*_1_>0) represents the manager’s green management skills (green management and coordination skills) and *η*(0<*η*<1) represents the extent to which the organization’s green atmosphere is effective. As *η* approaches 1, it means that the green atmosphere of the enterprise is more defective [51, 55], and *η* = 1 means the green atmosphere is fully effective in motivating employees to be green. On the contrary, a lower *η* means the green atmosphere of the enterprise is less effective, and it is difficult to motivate employees’ behaviors *e* represents the level of effort of the agents [77].When *e* is 0, effort costs do not occur when agents do not exert any effort and no effort cost is occurs. The larger the value of *e*, i.e., the greater the cost of the agent’s effort, the higher the consequent utility [78]. The performance of double carton targets implementation depends not only on the level of green management by GCG and green innovation behaviors by employees, but it is also influenced by external random variables. *θ* is a random disturbance term, with *θ*_1_ and *θ*_2_ representing the uncertainty risk factors encountered by GCG and employees, respectively, in implementing the double carton targets. It follows normal distribution *θ*_1_~(0,*σ*_1_^2^) and *θ*_2_~(0,*σ*_2_^2^). *σ*_1_ *and σ*_2_ are the green standard deviation, reflecting the degree of uncertainty in the performance outputs of the green innovation behaviors of managers and employees due to the influence of external random factors. Energy saving and emission reduction, as well as green innovative behaviors, are designed to enhance the environmental performance of the enterprise, and the high degree of uncertainty and difficulty in measuring environmental performance outputs are some of the difficulties that lead to the implementation of double carton targets in equipment manufacturing companies [79, 80].

Assumption 3:The cost of the agent’s efforts in the implementation of double carton targets is $C(e_{i})=\frac{1}{2}m_{i}{e_{i}}^{2}$ where *m*_*i*_ (*m*_*i*_>0, *i* = 1,2) is the corresponding cost factors for GCG and employees respectively, implying the level of effort cost of the respective green innovation behaviors.

Assumption 4: According to the contract of the proxy contract signed between the GCG and the employee, the employee receives a fixed income of remuneration component. Incentivized based on green performance outputs. Therefore, the GCG enters into a linear contract with employees, represented by *W*_2_ = *α*_2_+*β*_2_(*π*_2_) where *β*_2_(0≤*β*_2_≤1) represents the incentive intensity of the GCG, based on the environmental performance output.

The employee compensation income deducting the effort cost is the benefit function for green innovation behaviors.


$$u_{2}=W_{2}-C(e_{2})=a_{2}+\beta_{2}(\lambda_{2}e_{2}+\theta_{2})-\frac{1}{2}m_{2}{e_{2}}^{2}$$ (1)

For risk-averse employees, the cost of risk borne by employees is

$$RC_{2}=\frac{1}{2}\rho_{2}{\beta_{2}}^{2}{\sigma_{2}}^{2}$$ (2)

Their certainty of equivalent income CE2 is equal to their expected return minus the cost of risk (Eq 2) that the employee bears [5].

The employee’s deterministic equivalent income is:

$$CE_{2}=E(u_{2})-RC_{2}=a_{2}+\beta_{2}\lambda_{2}e_{2}-\frac{1}{2}m_{2}{e_{2}}^{2}-\frac{1}{2}\rho_{2}{\beta_{2}}^{2}{\sigma_{2}}^{2}$$ (3)

Assumption 5: According to the principal-agent contract signed by the general manager and the GCG. The fixed income of the green coordination team is *α*_1_, and it is motivated by the coefficient on the basis of the green performance output *β*_1_.Therefore, the general manager enters into a linear contract with the GCG, represented by *W*_1_ = *α*_1_+*β*_1_(*π*_1_). *W*_1_ represents the linear income of the manager. *α*_1_ is a fixed remuneration component. *β*_1_(0≤*β*_1_≤1) represents the incentive intensity of the general manager.

The income function of its GCG is remuneration income of the green coordination group minus the effort cost.

$$u_{1}=W_{1}-W_{2}-C(e_{1})=\alpha_{1}+\beta_{1}\pi_{1}-\alpha_{2}-\beta_{2}\pi_{2}-\frac{1}{2}m_{1}{e_{1}}^{2}$$ (4)

*u*_1_ represents the GCG’s actual return. For a risk-averse GCG, the cost of risk borne by the GCG is:

$$RC_{1}=\frac{1}{2}\rho_{1}({\beta^{2}}_{1}{\sigma_{1}}^{2}+{\beta_{2}}^{2}{\sigma_{2}}^{2})$$ (5)

The deterministic equivalent revenue CE1 is equal to its expected return minus the cost of risk, and the GCG’s certainty equivalent income is:

$$\begin{array}{l} CE_{1}=E(u_{1})-RC_{1}\\ =a_{1}+\beta_{1}\lambda_{1}e_{1}+\beta_{1}\eta \lambda_{2}e_{2}-a_{2}-\beta_{2}\lambda_{2}e_{2}-\frac{1}{2}m_{1}{e_{1}}^{2}-\frac{1}{2}\rho_{1}({\beta_{1}}^{2}{\sigma_{1}}^{2}+{\beta_{2}}^{2}{\sigma_{2}}^{2}) \end{array}$$ (6)

Assumption 6: The general manager’s deterministic equivalent income is the number of green benefits net of incentive costs resulting from the implementation of the double carbon targets. As the general manager is risk neutral, his determination of equivalent income is equal to the expected return, i.e.


$$E(u_{0})=-\alpha_{1}+(1-\beta_{1})(\lambda_{1}e_{1}+\eta \lambda_{2}e_{2})$$ (7)

The key parameters involved in this paper and their meanings are shown in **Table 1.**

**Table 1:** Main parameters and meanings.

Parameters	Meaning	Parameters	Meaning
*λ*_1_	Green management capability of managers	*λ*_2_	Employee behavior competence
*η*	Organizing a green atmosphere	*ρ*	Absolute risk size degree
*θ*	Environmental risk factor	*σ*	Green standard deviations
*e*_1_	The level of managerial effort in the implementation of the green strategy	*e*_2_	The level of employee involvement in the implementation of the green strategy
*m*_1_	Cost of effort factor for green management by managers	*m*_2_	Staff effort cost factor for green strategy implementation
*β*_1_	General manager green management incentive strength	*β*_2_	Managerial motivational intensity
*α*_1_	Fixed compensation for managers	*α*_2_	Fixed compensation for employees
CE1	Certainty equivalent income from green management for managers	CE_2_	Certainty equivalent income from employees’ green behaviors
*RC*_1_	The cost of risk borne by managers in green management	*RC*_2_	The cost of risk borne by employees in green management and meanings.

### 3.3 Model construction and solving

Green innovation behavioral incentives between managers and employees can be addressed as a planning issue, as follows:

$$\begin{array}{l} \;\underset{\alpha_{2},\;\beta_{2}}{\mathrm{Max}}\;{\mathrm{CE}}_{1}\\ (P1)\;s.t.\\ \;e_{2}\in \arg\;\max\;{\mathrm{CE}}_{2}\;(IC)\\ \;{\mathrm{CE}}_{2}\geq {\bar{\omega }}_{2}\;(IR) \end{array}$$

Solving the constraint shows that employees will choose ${e_{2}}^{*}=\frac{\beta_{2}\lambda_{2}}{m_{2}}$as their optimal level of effort and the GCG’s optimal choice is to pay the employee only an amount equal to his or her retained earnings.

Therefore, the constraint (P1) is taken as (IR), an equal sign, and substituted into the objective function, together with the constraint (IC), which solves *e*_2_ in the target function, thus eliminating *α* and *e*_2_, and obtaining the following equivalence problem (P2):

$$\begin{array}{l} \left(\mathrm{P2}\right)\\ \underset{\alpha_{2},\beta_{2}}{\mathrm{Max}}\;a_{1}+\beta_{1}(\lambda_{1}e_{1}+\eta \lambda_{2}\frac{\beta_{2}\lambda_{2}}{m_{2}})-\frac{1}{2}m_{1}{e_{1}}^{2}-\frac{{\beta_{2}}^{2}{\lambda_{2}}^{2}}{2m_{2}}-\frac{1}{2}\rho_{1}({\beta_{1}}^{2}{\sigma_{1}}^{2}+{\beta_{2}}^{2}{\sigma_{2}}^{2})-\frac{1}{2}\rho_{2}{\beta_{2}}^{2}{\sigma_{2}}^{2}-{\bar{\omega }}_{2} \end{array}$$

The solution to (P2) is as follows:

$$\beta_{2}^{*}=\frac{\beta_{1}{\lambda_{2}}^{2}\eta }{{\lambda_{2}}^{2}+m_{2}{\sigma_{2}}^{2}(\rho_{1}+\rho_{2})}$$ (8)

$$e_{2}^{*}=\frac{\beta_{1}{\lambda_{2}}^{3}\eta }{m_{2}({\lambda_{2}}^{2}+m_{2}{\sigma_{2}}^{2}(\rho_{1}+\rho_{2}))}$$ (9)

The incentive for green innovation behaviors between the general manager and the GCG can be seen as a planning issue, as follows (P3):

$$\begin{array}{l} \;\underset{\alpha_{1},\;\beta_{1}}{\mathrm{Max}}\;\alpha_{1}+(1-\beta_{1})(\lambda_{1}e_{1}+\eta \lambda_{2}e_{2})\\ (P3)\;s.t.\\ \;e_{1}\in \arg\;\max\;{\mathrm{CE}}_{1}\;(IC_{1})\\ \;{\mathrm{CE}}_{1}\geq {\bar{\omega }}_{1}\;(IR_{1}) \end{array}$$

By solving the argument of maxima of (IC_1_) in problem (P3), we conclude that a GCG’s optimal effort level is ${e_{1}}^{*}=\frac{\beta_{1}\lambda_{1}}{m_{1}}$. The general manager’s optimal choice is to pay the GCG an amount equal to the reserve level salary. We substitute this into the objective function *e*_1_ together with the constraint (IC_1_) solved previously, thus eliminating *α*_1_ and *e*_1_, and obtaining the equivalence problem (P4).


$$\begin{array}{l} \left(P4\right)\;\underset{\alpha_{1},\beta_{1}}{\mathrm{Max}}-{\bar{\omega }}_{1}-{\bar{\omega }}_{2}-\frac{{\beta_{1}}^{2}\eta^{2}{\lambda_{2}}^{6}}{2m_{2}{\left({\lambda_{2}}^{2}+m_{2}{\sigma_{2}}^{2}(\rho_{1}+\rho_{2})\right)}^{2}}-\frac{{\beta_{1}}^{2}{\lambda_{2}}^{4}\rho_{2}\eta^{2}{\sigma_{2}}^{2}}{2{\left({\lambda_{2}}^{2}+m_{2}{\sigma_{2}}^{2}(\rho_{1}+\rho_{2})\right)}^{2}}\\ -\frac{{\lambda_{1}}^{2}{\beta_{1}}^{2}}{2m_{1}}-\frac{1}{2}\rho_{1}{\sigma_{1}}^{2}{\beta_{1}}^{2}-\frac{{\beta_{1}}^{2}{\lambda_{2}}^{4}\rho_{1}\eta^{2}{\sigma_{2}}^{2}}{2{\left({\lambda_{2}}^{2}+m_{2}{\sigma_{2}}^{2}(\rho_{1}+\rho_{2})\right)}^{2}}+\frac{\beta_{1}{\lambda_{1}}^{2}}{m_{1}}+\frac{\beta_{1}{\lambda_{2}}^{4}\eta^{2}}{m_{2}({\lambda_{2}}^{2}+m_{2}{\sigma_{2}}^{2}(\rho_{1}+\rho_{2}))} \end{array}$$

The solution of (P4) is:

$${\beta_{1}}^{*}=\frac{m_{2}{\lambda_{1}}^{2}({\lambda_{2}}^{2}+m_{2}{\sigma_{2}}^{2}(\rho_{1}+\rho_{2}))+m_{1}\eta^{2}{\lambda_{2}}^{4}}{m_{2}{\lambda_{1}}^{2}({\lambda_{2}}^{2}+m_{2}{\sigma_{2}}^{2}(\rho_{1}+\rho_{2}))+m_{1}\eta^{2}{\lambda_{2}}^{4}+m_{1}m_{2}({\lambda_{2}}^{2}+m_{2}{\sigma_{2}}^{2}(\rho_{1}+\rho_{2}))\rho_{1}{\sigma_{1}}^{2}}$$ (10)

$${e_{1}}^{*}=\frac{m_{2}{\lambda_{1}}^{3}({\lambda_{2}}^{2}+m_{2}{\sigma_{2}}^{2}(\rho_{1}+\rho_{2}))+m_{1}\eta^{2}\lambda_{1}{\lambda_{2}}^{4}}{m_{1}m_{2}{\lambda_{1}}^{2}({\lambda_{2}}^{2}+m_{2}{\sigma_{2}}^{2}(\rho_{1}+\rho_{2}))+{m_{1}}^{2}\eta^{2}{\lambda_{2}}^{4}+{m_{1}}^{2}m_{2}({\lambda_{2}}^{2}+m_{2}{\sigma_{2}}^{2}(\rho_{1}+\rho_{2}))\rho_{1}{\sigma_{1}}^{2}}$$ (11)

## 4. Results

### 4.1 Impact of model parameters on managers’ effort and incentive coefficients in green strategy implementation

**Proposition 1**: In Eq (10), the optimal green incentive coefficient (intensity) of the general manager towards the manager $\beta_{1}^{*}$ depends on the parameters *λ*_1_, *m*_1_, *ρ*_1_ and $\sigma_{1}^{2}$.

We find the first-order derivatives of *λ*_1_, *m*_1_, *ρ*_1_ and $\sigma_{1}^{2}$ with respect to $\beta_{1}^{*}$ in Eq (10).


$$\frac{\partial {\beta_{1}}^{*}}{\partial \lambda_{1}}=\frac{2m_{1}{m_{2}}^{2}\lambda_{1}y\rho_{1}{\sigma_{1}}^{2}}{{\left(m_{2}{\lambda_{1}}^{2}y+m_{1}\eta^{2}{\lambda_{2}}^{4}+m_{1}m_{2}y\rho_{1}{\sigma_{1}}^{2}\right)}^{2}}>0$$ (12)

$$\frac{\partial {\beta_{1}}^{*}}{\partial m_{1}}=-\frac{{m_{2}}^{2}{\lambda_{1}}^{2}y\rho_{1}\sigma_{1}^{2}}{{\left(m_{2}{\lambda_{1}}^{2}y+m_{1}\eta^{2}{\lambda_{2}}^{4}+m_{1}m_{2}y\rho_{1}{\sigma_{1}}^{2}\right)}^{2}}<0$$ (13)

$$\frac{\partial {\beta_{1}}^{*}}{\partial \rho_{1}}=\frac{-m_{1}{m_{2}}^{2}{\lambda_{1}}^{2}y^{2}{\sigma_{1}}^{2}-{m_{1}}^{2}m_{2}{\lambda_{2}}^{4}y\eta^{2}{\sigma_{1}}^{2}-{m_{1}}^{2}{m_{2}}^{2}{\lambda_{2}}^{4}\eta {\sigma_{1}}^{2}{\sigma_{2}}^{2}\rho_{1}}{{\left(m_{2}{\lambda_{1}}^{2}y+m_{1}\eta^{2}{\lambda_{2}}^{4}+m_{1}m_{2}y\rho_{1}{\sigma_{1}}^{2}\right)}^{2}}<0$$ (14)

$$\frac{\partial {\beta_{1}}^{*}}{\partial {\sigma_{1}}^{2}}=\frac{-m_{1}m_{2}y\rho_{1}}{{\left(m_{2}{\lambda_{1}}^{2}y+m_{1}\eta^{2}{\lambda_{2}}^{4}+m_{1}m_{2}y\rho_{1}{\sigma_{1}}^{2}\right)}^{2}}<0$$ (15)

Eq (12) shows that $\beta_{1}^{*}$ is positively correlated with *λ*_1_. Eqs (13), (14) and (15) show that there is a negative correlation of $\beta_{1}^{*}$ with *m*_1_, *ρ*_1_ and $\sigma_{1}^{2}$.

The optimal green management incentives designed by the general manager for managers are positively correlated with the managers’ ability to coordinate green initiatives [81]. Conversely, these incentives are negatively associated with the variance in the random variables of the managers’ effort cost factor, risk aversion, and environmental uncertainty. As such, increasing the intensity of green incentives allows companies to recruit managers with stronger potential for green management and coordination. This approach also motivates managers with lower effort cost coefficients (indicating management talent and effective communication skills) to engage more actively in green management, thereby enhancing environmental performance. Additionally, a lower variance in the random variables of environmental uncertainty leads to a stronger correlation between the GCG’s efforts in energy saving, emission reduction, and green innovation management, and the resulting environmental benefits. These benefits are more closely linked to the managers’ green efforts than to random variables, accurately reflecting their effort levels. Consequently, incentives for green management encourage the GCG to invest greater effort in such initiatives.

**Proposition2:** $e_{1}^{*}$ is increasingly monotonically related to *λ*_1_, and decreasingly monotonically related to *m*_1_, *ρ*_1_and $\sigma_{1}^{2}$.

Since ${e_{1}}^{*}=\frac{\beta_{1}\lambda_{1}}{m_{1}}$, it is deduced that:

$$\frac{\partial {e_{1}}^{*}}{\partial \lambda_{1}}=\frac{1}{m}\cdot \frac{\partial {\beta_{1}}^{*}}{\partial \lambda_{1}}+\frac{{\beta_{1}}^{*}}{m}>0$$ (16)

$$\frac{\partial {e_{1}}^{*}}{\partial m_{1}}=\frac{\lambda_{1}}{m_{1}}\cdot \frac{\partial {\beta_{1}}^{*}}{\partial m_{1}}-\frac{\lambda_{1}\beta_{1}}{{m_{1}}^{2}}<0$$ (17)

$$\frac{\partial {e_{1}}^{*}}{\partial \rho_{1}}<0$$ (18)

$$\frac{\partial {e_{1}}^{*}}{\partial {\sigma_{1}}^{2}}<0$$ (19)

Eq (16) shows that $e_{1}^{*}$ is positively correlated with *λ*_1_. Eqs (17), (18) and (19) show that there is a negative correlation of $e_{1}^{*}$ with *m*_1_, *ρ*_1_ and $\sigma_{1}^{2}$.

Enterprises require GCGs to integrate and coordinate various resources and capabilities to promote the implementation of double carton targets, such that the more capable (higher *λ*_1_) managers have extensive green management experience and the ability to coordinate different parts of the enterprise to achieve green synergy; the less costly (lower *m*_1_) managers have a strong ability to adapt to a green environment and learn, and have the quality of agile management. Risk-averse managers (lower *ρ*_1_) are easily challenged by the implementation of green strategies and seek higher psychological and material rewards. As a result, GCGs who are more likely to behave in a way that reflects their own performance in the process of implementing a green strategy from the top down (lower $\sigma_{1}^{2}$) can be more motivated towards green management and coordination roles, and play a greater green role at the organizational level.

### 4.2 The effect of organizational green climate on the optimal motivation coefficient and employee effort

Proposition 3:

$\beta_{1}^{*}$, $e_{1}^{*}$, $\beta_{2}^{*}$ and $e_{2}^{*}$ are all positively correlated with *η*.

We find the first-order derivatives of $\beta_{1}^{*}$, $e_{1}^{*}$, $\beta_{2}^{*}$ and $e_{2}^{*}$ with respect to *η*.

$$\frac{\partial {\beta_{1}}^{*}}{\partial \eta }=\frac{2\eta y{m_{1}}^{2}m_{2}\rho_{1}{\sigma_{1}}^{2}{\lambda_{2}}^{4}}{{\left(m_{2}{\lambda_{1}}^{2}y+m_{1}\eta^{2}{\lambda_{2}}^{4}+m_{1}m_{2}y\rho_{1}{\sigma_{1}}^{2}\right)}^{2}}>0$$ (20)

$$\frac{\partial {e_{1}}^{*}}{\partial \eta }=\frac{\lambda_{1}}{m_{1}}\cdot \frac{\partial {\beta_{1}}^{*}}{\partial \eta }>0$$ (21)

$$\frac{\partial {\beta_{2}}^{*}}{\partial \eta }=\frac{{\lambda_{2}}^{2}}{y}({\beta_{1}}^{*}+\frac{\eta \partial {\beta_{1}}^{*}}{\partial \eta })>0$$ (22)

$$\frac{\partial {e_{2}}^{*}}{\partial \eta }=\frac{{\lambda_{2}}^{3}}{m_{2}y}({\beta_{1}}^{*}+\frac{\eta \partial {\beta_{1}}^{*}}{\partial \eta })>0$$ (23)

Organizational green climate refers to the green climate created by the implementation of a set of systems and policies (environmental policies, practices and procedures, etc.) that contribute to the achievement of sustainable development. Enterprises create an organization’s green atmosphere by building green systems and policies that regulate design, production, marketing and other aspects, thus enhancing the unified green cognition within equipment manufacturing enterprises, improving the green awareness power of general managers [82], green resource allocation ability and the grasp of managers’ incentive emphasis, enhancing managers’ green management and coordination ability, improving green service awareness [83], and strengthening employees’ willingness to save energy and protect the environment and their green innovation, which in turn has a guiding effect on employees’ green innovation behaviors [6].

### 4.3 The effects of relevant parameters on the level of effort and incentive coefficient of employees’ green innovation behaviors

Proposition 4: $\beta_{2}^{*}$ is positively correlated with *λ*_1_ and *λ*_2_, while $\beta_{2}^{*}$ is negatively correlated with *m*_1_, *ρ*_1_, $\sigma_{1}^{2}$, *m*_2_, *ρ*_2_ and $\sigma_{2}^{2}$.

We find the first-order derivatives of *λ*_1_, *m*_1_, *ρ*_1_ and $\sigma_{1}^{2}$ with respect to $\beta_{2}^{*}$ via Eq (7).


$$\frac{\partial {\beta_{2}}^{*}}{\partial \lambda_{1}}=\frac{{\lambda_{2}}^{2}\eta }{{\lambda_{2}}^{2}+m_{2}{\sigma_{2}}^{2}(\rho_{1}+\rho_{2})}\cdot \frac{2m_{1}{m_{2}}^{2}\lambda_{1}y\rho_{1}{\sigma_{1}}^{2}}{{\left(m_{2}{\lambda_{1}}^{2}y+m_{1}\eta^{2}{\lambda_{2}}^{4}+m_{1}m_{2}y\rho_{1}{\sigma_{1}}^{2}\right)}^{2}}>0$$ (24)

$$\frac{\partial {\beta_{2}}^{*}}{\partial m_{1}}=\frac{-{m_{2}}^{2}{\lambda_{1}}^{2}{\lambda_{2}}^{2}y\rho_{1}\sigma_{1}^{2}\eta }{({\lambda_{2}}^{2}+m_{2}{\sigma_{2}}^{2}(\rho_{1}+\rho_{2})){\left(m_{2}{\lambda_{1}}^{2}y+m_{1}\eta^{2}{\lambda_{2}}^{4}+m_{1}m_{2}y\rho_{1}{\sigma_{1}}^{2}\right)}^{2}}<0$$ (25)

$$\begin{array}{l} \frac{\partial {\beta_{2}}^{*}}{\partial \rho_{1}}=\frac{(-m_{1}{m_{2}}^{2}{\lambda_{1}}^{2}y^{2}{\sigma_{1}}^{2}-{m_{1}}^{2}m_{2}{\lambda_{2}}^{4}y\eta^{2}{\sigma_{1}}^{2}-{m_{1}}^{2}{m_{2}}^{2}{\lambda_{2}}^{4}\eta {\sigma_{1}}^{2}{\sigma_{2}}^{2}\rho_{1}){\lambda_{2}}^{2}\eta }{{\left(m_{2}{\lambda_{1}}^{2}y+m_{1}\eta^{2}{\lambda_{2}}^{4}+m_{1}m_{2}y\rho_{1}{\sigma_{1}}^{2}\right)}^{2}({\lambda_{2}}^{2}+m_{2}{\sigma_{2}}^{2}(\rho_{1}+\rho_{2}))}\\ -\frac{{\lambda_{2}}^{2}\eta \beta_{1}}{{\left({\lambda_{2}}^{2}+m_{2}{\sigma_{2}}^{2}(\rho_{1}+\rho_{2})\right)}^{2}}<0 \end{array}$$ (26)

$$\frac{\partial {\beta_{2}}^{*}}{\partial {\sigma_{1}}^{2}}=\frac{-m_{1}m_{2}y\rho_{1}}{{\left(m_{2}{\lambda_{1}}^{2}y+m_{1}\eta^{2}{\lambda_{2}}^{4}+m_{1}m_{2}y\rho_{1}{\sigma_{1}}^{2}\right)}^{2}}\cdot \frac{{\lambda_{2}}^{2}\eta }{{\lambda_{2}}^{2}+m_{2}{\sigma_{2}}^{2}(\rho_{1}+\rho_{2})}<0$$ (27)

All the relevant factors affecting the degree of the green motivation of GCG by general managers affect the degree of green innovation behaviors of management towards employees, in addition to similar coefficients affecting the degree of motivation of managers towards employees in the same direction. The incentive system is complex, with each component affecting each other and the whole body. Therefore, the construction of a green incentive system plays an important role in the implementation of double-carton targets.

Proposition 5: Employee effort in green innovation behaviors is positively correlated with *λ*_1_, and *λ*_1_ is negatively correlated with *m*_1_, *ρ*_1_, $\sigma_{1}^{2}$, *m*_2_, *ρ*_2_ and $\sigma_{2}^{2}$.

From ${e_{2}}^{*}=\frac{\beta_{2}\lambda_{2}}{m_{2}}$, it can be seen that the level of employee effort in energy conservation and green innovation is positively correlated with the intensity of managerial incentives for green innovation behaviors and the effectiveness of employee effort, while the cost of employee effort is negatively correlated with it. From ${e_{2}}^{*}=\frac{\beta_{1}{\lambda_{2}}^{3}\eta }{m_{2}y}$, it can be seen that the level of energy saving and green innovation effort of employees is also related to the level of optimal green motivation of the general manager to the GCG, and all factors that influence this are related to one another. For example, the level of green management shown by managers is positively correlated with the level of effort shown by employees. The higher the level of green management, the more the environment is improved for employees to be motivated to work green, which in turn converts their green intentions into behaviors [84].

## 5. Numerical analysis

Based on Propositions 1–5, this section uses MATLAB2016a software to develop a corresponding numerical simulation to extend the analysis. According to the principal-agent model, the initial parameter values are set for simulation analysis. This paper draws on the relevant academic literature on principal-agent modelling in order to establish the necessary parameters. Data for this study was obtained through a combination of expert interviews in the field of green development and the distribution of questionnaires. The questionnaire was primarily designed to assess the green management and coordination abilities of corporate managers, the green behavioral capabilities of employees, the effort costs for both managers and employees, the establishment of a green atmosphere, the risk preferences of managers, and the incentive situation. Following the collection of the questionnaires and the associated data, the initial assignments were determined by considering the green practices implemented by manufacturing companies. So, the model values are set as follows: *λ*_1_ = 1, *m*_1_ = 0.8, *ρ*_1_ = 0.5, $\sigma_{1}^{2}=3$, *λ*_2_ = 0.9, *m*_2_ = 0.3, *ρ*_2_ = 0.4, $\sigma_{2}^{2}=4$ and *η* = 0.8. When describing the variation of a parameter within a certain valid range, the other parameters are assumed to remain constant, and the graphs in Figs 2–10 are plotted to reflect the relationship between the parameters *λ*_1_, *λ*_2_, *m*_1_, *m*_2_, $\sigma_{1}^{2}$, $\sigma_{2}^{2}$, *ρ*_1_, *ρ*_2_, *η*, *β*_1_ and *β*_2_, respectively.

**Fig 2:** Relationship of *λ*_1_ with *β*_1_, *β*_2_, *e*_1_ and *e*_2_.

**Fig 3:** Relationship of *λ*_2_ with *β*_1_, *β*_2_, *e*_1_ and *e*_2_.

**Fig 4:** Relationship of *m*_1_ with *β*_1_, *β*_2_, *e*_1_ and *e*_2_.

**Fig 5:** Relationship of *m*_2_ with *β*_1_, *β*_2_, *e*_1_ and *e*_2_.

**Fig 6:** Relationship of $\sigma_{1}^{2}$ with *β*_1_, *β*, *e*_1_ and *e*_2_.

**Fig 7:** Relationship of $\sigma_{2}^{2}$ with *β*_1_, *β*_2_, *e*_1_ and *e*_2_.

**Fig 8:** Relationship of *ρ*_1_ with *β*_1_, *β*_2_, *e*_1_ and *e*_2_.

**Fig 9:** Relationship of *ρ*_2_ with *β*_1_, *β*_2_, *e*_1_ and *e*_2_.

**Fig 10:** Relationship of *η* with *β*_1_, *β*_2_, *e*_1_ and *e*_2_.

Fig 2 shows that there is a positive correlation between GCG’ green management ability *λ*_1_ and *β*_1_, *β*_2_, *e*_1_, *e*_2_. When the management and coordination capacity of the GCG is weak, the general manager increases the intensity of the incentive, the GCG rapidly puts in more effort, and the incentive effect increases. The GCG’s capacity is enhanced, which means that the enterprise has a good green atmosphere, the whole business process involves a better allocation of green resources, and the employees implement energy saving, emission reduction and green innovation behaviors. However, when the GCG’s green management and coordination capacity reaches a certain threshold, the level of effort of the GCG and employees does not rise as quickly as the intensity of the incentive increases. At this point, the general manager’s incentive effect on the green coordination team tends to level off.

Fig 3 shows that there is a positive correlation between employees’ ability to act green *λ*_2_ and *β*_1_, *β*_2_, *e*_1_, *e*_2_. Firstly, when the staff’s ability to act green is weak, the incentive measures of the GCG that stimulate staff to enhance their awareness of energy saving, environmental protection and green innovation increase the staff’s efforts in a linear fashion, with a significant incentive effect. When the incentive intensity of the GCG reaches a certain value, the incentive effect increases at a slower rate. In enterprises, the strength of employees’ green innovation behaviors also affects the general manager’s incentive intensity towards the GCG, and the level of effort of the GCG. When the employees’ level of green innovation behavioral competence is low, the general manager increases the incentive intensity of the GCG and raises its competence level, with the aim of influencing employees’ green innovation behavioral competence and implementing the green strategy efficiently. Therefore, the general manager and the GCG work together to build a green organizational atmosphere, develop green techniques, and pass on their skills to enhance employees’ organizational green identity, improve their green competencies and their level of effort, and thus positively develop the level of effort of employees. Figs 2 and 3 together illustrate that incentives for managers should be developed with consideration of their capabilities and needs and the effect they have on the level of effort of employees. In contrast, the design of incentives for employees does not take into account their ability to work hard for their superiors, their ability to control them, or the size of the incentive–cost ratio.

Fig 4 shows that there is a decreasing trend amongst *β*_1_, *β*_2_, *e*_1_, *e*_2_ in the cost of the managerial effort factor as *m*_1_ increases. The GCG increases the knowledge and experience of green management, builds and runs an organizational green climate, and motivates employees to reduce the negative effects. When the cost of green management and coordination effort is low, the GCG encounters less resistance in carrying out green management tasks, the environmental performance is more effective, and the green coordination team is more willing to put in more effort. When the cost of effort of the GCG reaches a certain value, it means that the GCG has encountered bottlenecks in carrying out its management tasks. For example, in the process of digital transformation, how the GCG should coordinate the allocation of green resources and obtain national green certification is a key issue. The level of effort of the GCG will at this point rapidly decline, or they may even choose to give up. At this point, the general manager needs to adjust the incentive contract to increase the level of effort by means of additional training and moral incentives, in order to guarantee the implementation of the green strategy and the development of the coordination team’s sense of self-worth.

The range of values *m*_2_ chosen for Fig 5 is between 0 and 0.5, because it is only when this range is used that the trend of the four lines can be clearly distinguished.

When the cost of employee effort towards green innovation behaviors is low, it signifies a minimal negative impact from learning and sharing green knowledge, and exerting effort in energy saving and green innovation. Under these conditions, employees are more inclined to increase their efforts in improving green innovation capabilities. However, as the negative impact of employee effort escalates, the GCG becomes the first to notice obstacles in implementing green management, leading to a reduction in their own effort level. Consequently, at a certain threshold, employees’ efforts diminish significantly. Therefore, it is advisable to maintain the GCG’s incentive range until this threshold is reached. Beyond this point, the GCG should consider terminating the contract and instead utilize psychological contracts, moral incentives, and green training to transform employees’ willingness to adopt green practices into sustained green innovation behaviors.

The integrated examination of Figs 4 and 5 illustrates that, for the GCG, a low cost of effort results in heightened exertion, driven by incentives form the general manager. This dynamic also extends to encouraging employees to adopt green behavior. Conversely, form employees’ perspective, as the cost of effort reaches a certain, the GCG perceives the impact and subsequently diminishes its effort. This, in turn prompts employees to reduce or discontinue their green innovation behaviors. Consequently, the general manager delineates the range and level of incentives based on the uncertainty and effort cost encountered by the GCG in attaining the double carbon targets.

Figs 6 and 7 illustrate that heightened uncertainty concerning shifts in both the internal and external green landscape can impede the translation of the Green Corporate Governance’s (GCG) management endeavors into tangible green performance outcomes. Consequently, a decision may be made to scale back the level of effort. This decision, in turn, influences the effort level of the employees, leading to a precipitous decline in their green innovation initiatives, thereby significantly compromising the efficacy of implementing the dual carbon targets across the organization. Notably, as employees encounter escalating uncertainty regarding their green environment, their individual green endeavors experience a rapid decline, underscoring their heightened sensitivity to uncertainty. In contrast, fluctuations in management effort plateau, subsequently stabilizing the level of management incentive. Hence, it becomes imperative for the general manager to calibrate management incentives in a manner that considers potential increases in either the proportional or absolute magnitude of incentive costs, or alternatively, to supplement with more nuanced implicit incentives, such as psychological contracts and fostering an organizational climate conducive to green initiatives [79].

Fig 8 illustrates that when the GCG exhibits greater risk tolerance and adeptly navigates green uncertainty, the general manager delegates a higher volume of green management tasks. These tasks encompass the coordinating of resources across design, production, marketing and other processes, aiming to foster agile management and bolster the enterprise’ s green output of Conversely, as the GCG’S risk tolerance diminishes, the general manager encounters challenges in utilizing contractual incentives to elevate the effort levels of both the GCG and employees. The level of certainty surrounding green strategy implementation becomes paramount. Consequently, in the selection and formation of the GCG, the general manager prioritizes individuals inclined towards risk-taking and engagement in green and innovative endeavors. This strategic approach aims to optimize green performance while nurturing employees’ commitment go green values.

Fig 9 illustrates that, firstly, the uncertainty of the green performance resulting from energy saving and environmental behavior is so high that employees who prefer risk are more likely to be motivated by green innovation activities, while those with a weak risk tolerance are likely to choose inaction. Secondly, a reduction in employees’ ability to take risks not only reduces their own optimal incentive strength, but also negatively affects the optimal incentive strength of the green coordination team, while the magnitude of the change between the two tends to be balanced. General manager and GCG select employees who have a preference for risk.

Fig 10 shows that the GCG creates a green atmosphere through the systems and policies that govern the implementation of the double carton targets in enterprises. As the influence of the green atmosphere grows, the GCG and employees develop a unified perception of greenness and increase their respective levels of effort. The GCG is motivated by the general manager to make more management and coordination efforts to ensure the effectiveness of the double carton targets, and to build and improve the organization’s green atmosphere. The more effective the green climate is, the more the GCG will be able to motivate employees without increasing their incentives, and the more their green capabilities will develop.

In compared to prior studies, this paper holds significant theoretical and practical implications. Previous research on employees’ environmental behavior mainly focuses on the individual [80]and organizational levels [81], yet no one have integrated both within a unified framework. Leveraging the dual principal-agent model, this study incorporates the green innovation behavior of employees and GCG into a cohesive to analyze influencing factors and pathways. The finding that employees inclined towards risk exhibit a higher propensity for engagement in green innovation activities corroborates findings from studies on the effects of equity incentive [82, 83]. Previous investigated have examined enterprise employees’ green training and consensus from the standpoint of organizational climate [50]. Drawing from the double principal-agent theory, this paper delves into the pertinent research regarding the GCG’s establishment of a green organizational climate and its on employee effort level, with findings aligning [85–87].

## 6. Conclusions and practical implications of the study

### 6.1 Conclusions

The innovative behavior exhibited by employees holds paramount importance for equipment manufacturing enterprises, facilitating the reduction of energy consumption, environmental preservation, and the production of green products or provision of green services. Consequently, this paper endeavors to investigate strategies for motivating employees to enhance their awareness of green behavior and advance research on participation in green environmental protection initiatives. Leveraging the dual principal-agent theory, a dual principal-agent model is formulated, focusing on the following four aspects for study and elucidation.

1. The optimal incentive coefficient for green innovation behaviors, as determined by the general manager, exhibits a positive correlated with the GCG’s green management capability. Conversely, it demonstrates a negatively correlation with factors such as the GCG’s effort cost, risk aversion, and green variance. Within a specific threshold, augmenting the incentive for green innovation behaviors proves effective in enhancing the efforts of both the GCG and employees. However, surpassing this threshold results in diminishing, rendering further increases in incentive intensity ineffective.
2. The cost of GCG effort exhibits an inverse relationship with the general manager’s incentive for green innovation behaviors, the GCG’s incentive factor, and the efforts of both the GCG and employees. A less pronounced negative impact of the GCG’s effort results in a more substantial incentive effect. When the cost of GCG effort escalates to a certain level, There is a risk of inactivity. In such cases, enterprises should contemplate suspending contractual approaches and explore alternative methods to ensure the continued implementation of green innovation behaviors and unlock the full potential of the coordination team.
3. The risk aversion exhibited by both the GCG and employees, coupled with environmental uncertainty, demonstrates a negative correlation with the general manager’s incentive for green innovation behaviors, the GCG’s incentive factor, and the effort levels of the GCG and employees. Elevated risk aversion and a more conducive external environment for green innovation behaviors contribute to heightened effort from the GCG and employees, thereby increasing the likelihood of improved performance in green innovation behaviors.
4. The GCG fosters a green organizational climate that amplifies the effort levels in employees’ green innovation behaviors as well as their individual contributions. Green policies and regulations aid in fostering a consensus among enterprise employees regarding green practices, consequently enhancing green performance. Within a positive green organizational climate, the output of performance in green innovation behaviors remains significant, even in scenarios where employee motivation levels are low.
5. Employee green behavior significantly impacts an organization’s environmental performance, resulting in cost savings, decreased environmental impact, and improved public perception. Hence, it is imperative for organizations to foster green behaviors among their workforce through education, incentives, and robust environmental policies.

To cultivate a green organizational climate, manufacturing companies can implement the following measures::

Firstly, articulate the environmental attitudes and preferences of company executives and establish corresponding incentives levels. This clarity will empower employees to comprehend the anticipated of their efforts towards green behavior.

Secondly, institute and refine the green management system. This entails the implementation of green supply chain management, environmental management systems, and energy-saving and emission reduction systems. By defining explicit goals for the implementation of green strategy and delineating corresponding responsibilities, companies can stimulate the formation of a green coordination team, fostering active engagement from employees in the enterprise’s green strategy implementation.

Thirdly, it is imperative to implement green training initiatives. Manufacturing enterprises ought to provide tailored green training programs encompassing topics such as environmental consciousness, energy conservation techniques, emission reduction strategies, and awareness of green innovation. This comprehensive training regimen will serve to enhance employees’ environmental awareness, bolster their commitment to sustainable practices, refine their proficiency in green technologies, and facilitate their proactive engagement in green innovation endeavors. With the growing integration of digital technology, the shift towards flatter organizational structures, and the heightened levels of both horizontal and vertical communication within companies, there is a rising challenge in designing incentives for green innovation behaviors. The perspectives presented in this paper propose innovative approaches for developing incentive mechanisms that not only encourage green innovation behaviors among employees but also cultivate a mutually beneficial relationship between employees and the organization.

To effectively devise green innovation incentive mechanisms customized to diverse employee characteristics, companies may contemplate the following strategies:

1. Tailored Incentive Programs: Formulate incentive schemes that accommodate the distinct characteristics and preferences of individual employees. For example, younger employees may be motivated by prospects for skill development and career advancement, while older employees may place greater importance on acknowledgment and financial rewards.
2. Performance-Based Rewards: Introduce performance-based incentives that recognize and reinforce green innovation endeavors. This may involve bonuses, promotions, or other tangible rewards for employees demonstrating a steadfast commitment to sustainable practices and green innovation.
3. Green Training and Development: Offer comprehensive green training programs to empower employees with the requisite knowledge and skills for green innovation. These initiatives may encompass workshops, seminars, and certifications concentrating on sustainability, energy efficiency, waste reduction, and other relevant areas.
4. Atmosphere Building: Cultivate a positive and supportive work environment conducive to fostering creativity, risk-taking, and experimentation in green innovation. This entails promoting open communication, acknowledging achievements, and providing resources to support employees in developing their green initiatives.

### 6.2 Practical implications of the study

This study utilizes the double principal-agent theory to investigate the incentives of general managers and Green Coordination Groups (GCG), as well as the green innovation behaviors of enterprise employees. The findings contribute to enriching the theoretical comprehension of employee-driven green innovation and provide practical insights to improve the efficacy of green strategy implementation in enterprises., there by fostering high-quality development.

1. For equipment manufacturing enterprises, the establishment and cultivation of a green coordination team with robust green innovation capabilities are paramount. The dual carbon target represents a multifaceted strategy that requires a delicate balance between meeting customer demands and economic performance while prioritizing energy conservation, environmental protection, and the attainment of environmental performance objectives. This necessitates collaborative efforts across various dimensions. Furthermore, as most enterprises undergo digital transformation, the integration of digital technology has facilitated the adoption of flatter organizational structures. This dual organizational paradigm demands both horizontal inter-departmental synergy and vertical coordination at the employee level. In this context, the green coordination skills of managers play a pivotal role in the success of green innovation initiatives. The stronger the green management and coordination capabilities of the Green Coordination Group (GCG), the more emphasis is placed on green innovation behaviors within the team, leading to enhanced environmental performance of the enterprise at an accelerated pace. Consequently, the selection and recruitment of a green coordination team proficient in green innovation, the establishment and maintenance of a green-friendly atmosphere, and the encouragement of employees’ green consciousness exert a significant positive influence on the adoption of green innovation behaviors.
2. Providing guidance to the general manager on incentive design and implementation is paramount. The efficacy of incentives provided by the general manager to the Green Coordination Group (GCG) correlates positively with their level. Incentive intensity and measures should be customized based on the green management and coordination capabilities of the GCG. For example, when the GCG’s efforts reach a plateau, additional measures such as psychological contracts and vocational training should be utilized to sustain the effectiveness of incentives.
3. It is imperative to aid equipment manufacturing enterprises in devising effective combinations of green innovation incentives. Incentives have a profound impact on the level of green effort exerted by both the Green Coordination Group (GCG) and employees. A well-structured incentive framework strikes a balance between the interests and obligations of all parties involved. The double principal-agent approach entails designing incentives that are mutually agreeable to all stakeholders. Without this alignment, effective management becomes elusive, potentially compromising the objectives of green strategy implementation. The incentive package should be tailored to reflect the characteristics and capabilities of the GCG and employees in their green innovation endeavors. Notably, the general manager’s overarching design is crucial for attaining the enterprise’s dual carbon targets, necessitating ongoing adjustments to incentives based on the environmental performance of the GCG and the green innovation behaviors of employees. Thus, the general manager’s role in motivating the GCG’s green innovation behaviors is increasingly pivotal in enhancing the efficacy of the green strategy.

## 7. Limitations and future studies

### 7.1 Limitations

This study acknowledges several limitations in researching the dual principal-agent incentive model involving the general manager, green coordination team, and employees in manufacturing enterprises. These limitations stem from factors such as the assumptions underlying the application, the scope of the study, and constraints related to empirical data collection. For instance, the growing integration of digital technology and the establishment of a dedicated Green Coordination Team are pivotal considerations. This team plays a vital role in allocating both internal and external resources, which are essential for the effective implementation of the green strategy and serve as the groundwork for implementing dual agency incentives.

### 7.2 Futures studies

Firstly, the scope of responsibilities for Green Coordination Groups (GCG) within enterprises extends beyond mere green management to encompass the daily oversight of green innovation behaviors, which may involve addressing challenges such as raw material shortages. Subsequent research endeavors could delve into how managers and employees proficiently allocate resources to optimize these behaviors.

Secondly, although this paper concentrates on the implementation of dual carbon targets in enterprises and delineates various incentives for encouraging employee engagement in green innovation behaviors, it acknowledges the presence of additional influencing factors. These factors encompass societal attitudes towards energy conservation, knowledge of environmental protection, government regulations, incentives for green practices, and the influence of green human resource management within enterprises. Given the significance of these aspects in shaping employees’ green innovation behaviors, further investigation is warranted.

## Supporting information

S1 File (DOC)
